The article "Primum non nocere; It’s time to consider altitude training as the medical intervention it actually is!" was published in 2022. Journal: Front Psychol.

# Primum non nocere; It’s time to consider altitude training as the medical intervention it actually is!

**DOI:** 10.3389/fpsyg.2022.1028294

**Published:** 2022-12-13

**Authors:** Jeroen Van Cutsem, Nathalie Pattyn

**Affiliations:** ^1^Vital Signs and Performance Monitoring (VIPER) Research Unit, Royal Military Academy, Brussels, Belgium; ^2^Human Physiology and Sports Physiotherapy Research Group, Vrije Universiteit Brussel, Brussels, Belgium

**Keywords:** endurance, team-sport, performance, hypoxia, sleep, periodic breathing, physical activity, genetic polymorphisms

## Abstract

Sleep is one of the most important aspects of recovery, and is known to be severely affected by hypoxia. The present position paper focuses on sleep as a strong moderator of the altitude training-response. Indeed, the response to altitude training is highly variable, it is not a fixed and classifiable trait, rather it is a state that is determined by multiple factors (e.g., iron status, altitude dose, pre-intervention hemoglobin mass, training load, and recovery). We present an overview of evidence showing that sleep, and more specifically the prolonged negative impact of altitude on the nocturnal breathing pattern, affecting mainly deep sleep and thus the core of physiological recovery during sleep, could play an important role in intra- and interindividual variability in the altitude training-associated responses in professional and recreational athletes. We conclude our paper with a set of suggested recommendations to customize the application of altitude training to the specific needs and vulnerabilities of each athlete (i.e., primum non nocere). Several factors have been identified (e.g., sex, polymorphisms in the TASK2/KCNK5, NOTCH4 and CAT genes and pre-term birth) to predict individual vulnerabilities to hypoxia-related sleep-disordered breathing. Currently, polysomnography should be the first choice to evaluate an individual’s predisposition to a decrease in deep sleep related to hypoxia. Further interventions, both pharmacological and non-pharmacological, might alleviate the effects of nocturnal hypoxia in those athletes that show most vulnerable.

## Introduction

Elite athletes are constantly aiming to improve their performance, and eventually outperform their opponents. In this endeavor, various methods have been designed to gain an advantage over the other competitors. One of those methods, which has been in use for quite some time and remains very popular, is altitude training (Billaut et al., 2012; Girard et al., 2013; Nummela et al., 2021). Altitude training entered the world of sports science *via* endurance training. Ever since the 1960s, an escalation in the purposeful utilization of altitude to enhance endurance athletic performance has been observed (Balke et al., 1965). Traditionally, altitude training was organized so athletes simultaneously lived and trained at moderate natural altitude [i.e., hypobaric hypoxia; between ∼1,400 and 2,500 m above sea level (Mujika et al., 2019)]. Currently, multiple protocols of altitude training have been developed. A general distinction can be made between “live high, train high” (LHTH), “live high, train low” (LHTL), and “live low, train high” (LLTH) altitude training. The LHTL protocol is currently being put forward as the most effective one for training gains (Bonetti and Hopkins, 2009). In addition, the LLTH altitude training method is also gaining attention, as it can be applied with minimal costs and travel constraints for athletes (Girard et al., 2020). Several important features within these protocols are the type of hypoxic stimulus (i.e., normobaric or hypobaric), the hypoxic dose, the duration, the timing in the season, and the cumulative effect of multiple altitude training protocols [i.e., accumulated altitude training (Mujika et al., 2019)]. The ongoing research into the physiological mechanisms underpinning these, as well as the application of altitude training protocols, has resulted in altitude training not only being incorporated in every professional endurance athlete’s training program, but also being put forward as beneficial for team-sport athletes (Billaut et al., 2012; Aughey et al., 2013).

Turner et al. (2019) published a study on the perceptions of elite endurance athletes on the role and worth of altitude training. Elite British endurance runners (*n* = 39) and their support staff were surveyed prior to the 2012 Olympics Games. A total of 98% of the athletes and 95% of the support staff had utilized altitude and hypoxic training, or had advised it to athletes, and 75% of the athletes believed altitude and hypoxia to be a “very important” factor in their training regime (Turner et al., 2019). Moreover, camps lasting 3–4 weeks at 1,500–2,500 m were the most popular (Turner et al., 2019). Which is in conformity with research-based suggestions. In addition, a recent editorial of Girard (2022) emphasized the increasing interest in resistance training hypoxia (i.e., a LLTH-intervention). Deldicque (2022) reviewed sixteen original investigations that evaluated this LLTH-intervention and concluded that 2–3 sessions a week performed in hypoxic conditions for 4–6 weeks with simulated altitudes between 2,200 and 3,500 m should be recommended to individuals looking at potentiating the effects of resistance training.

The above shows that altitude training is still very popular and is applied in multiple ways within the sports community, and it demonstrates the strong conviction among athletes regarding its overall effectiveness to improve performance. This conviction of athletes is backed up by a significant amount of scientific data (Wilber, 2001; Bonetti and Hopkins, 2009; Gore et al., 2013; Mujika et al., 2019). Nonetheless, up to date, the efficacy of altitude training is still questioned by some, due the lack of rigorous and well-controlled investigations (Lundby et al., 2012; Lundby and Robach, 2016; Bejder and Nordsborg, 2018), and no scientific consensus exists. Since Lundby et al. (2012) published their critical views on the general application of altitude training to enhance performance in elite athletes, follow-up research has substantiated (Bejder et al., 2017; Robach et al., 2018; Racinais et al., 2021) these critical views of Lundby and colleagues. Nevertheless, the debate on the usefulness of altitude training in elite athletes is still ongoing (Millet et al., 2019), and currently revolves around whether athletes with an already high hemoglobin mass (i.e., elite athletes) can successfully increase their hemoglobin mass *via* altitude training. The hypoxia-induced increase in hemoglobin mass is the hematological mechanism that is thought to underly the positive impact of altitude training on endurance performance (Lundby et al., 2012), and is therefore pivotal in this whole discussion. Besides this mechanism, hypoxia-induced non-hematological mechanisms, such as mitochondrial gene expression and enhanced muscle buffering capacity have been described as well (Gore et al., 2007), but are less substantiated (Lundby et al., 2012). Based on the hematological mechanism, Lundby et al. (2012) suggested a differing impact of altitude training on elite and non-elite athletes. Non-elite athletes have a greater growth margin in their hemoglobin mass and therefore may experience more performance benefits from altitude training compared to elite athletes (Lundby et al., 2012). A suggestion that has been challenged lately by Millet et al. (2019). These authors are, based on their own analysis of the existing literature on LHTL studies including endurance athletes and reporting both initial values and percentage increase in hemoglobin mass measured with CO-rebreathing method and with a moderate typical error (<∼2%) for hemoglobin mass measurement, confident in supporting that the initial pre-LHTL hemoglobin mass value is of minimal importance (Millet et al., 2019).

As such, it seems that the discussion about the effectiveness of altitude training to trigger performance-improving adaptations has reached an impasse. A topic that could provide some new insights is the issue of intra- and interindividual variability in the response to altitude training, and the underlying mechanisms of these variabilities. Multiple studies have been performed that clearly outline the presence of both intra- and interindividual variability in the response to altitude training (Chapman et al., 1998; Friedmann et al., 2005; McLean et al., 2013a,b; Hauser et al., 2017; Nummela et al., 2021). Interindividual variability is variability, in this case in the response to altitude training, between individuals. While intraindividual variability is variability in a given individual in time. Intraindividual variability is per definition related to state-specific factors (e.g., iron status, training load, and recovery) that mediate the response to altitude training in a given individual. In contrast, interindividual variability can arise due to state-specific factors, which results in varying differences between individuals in time. Or, it can arise due to trait-specific factors (e.g., genetics), which results in replicable and robust differences in the response to altitude training between individuals in time. Of course, once stable interindividual variability is observed, the concept of responders and non-responders comes forward. Chapman et al. (1998) were the first to stress the possibility that being a responder or non-responder to altitude training might be a fixed genetic trait. However, this suggestion has been refuted by research including McLean et al. (2013a) and Nummela et al. (2021). These studies (McLean et al., 2013a; Nummela et al., 2021) have investigated the intra- and interindividual variability in the response to altitude training. The results clearly demonstrated that multiple state factors [e.g., iron status, altitude dose, pre-intervention hemoglobin mass, training load and recovery (Nummela et al., 2021)] moderated the responsiveness to altitude training. Subsequently, Nummela et al. (2021) concluded that the responsiveness to altitude training is not a fixed and classifiable trait. A conclusion that holds merit but that might be an oversimplification of the mechanisms underlying the observed variability, as trait influences cannot be discarded based on the presence of state-related intra- and interindividual variability. The determination and evaluation of all state and trait-specific factors that could influence an athlete’s response to altitude training is currently ongoing (McLean et al., 2013a; Nummela et al., 2021). Nummela et al. (2021) showed that the mean effectiveness of altitude training in yielding an increase in hemoglobin mass could rise from 56 to 69% when targeting altitude exposure (2,000–2,500 m), iron deficiency and inflammation as moderating state factors. This emphasizes the need to carefully consider all the possible moderating state factors that may influence an athlete’s response to altitude training. Furthermore, these findings stress the need for future research to describe more accurately how these different influencing state factors (and potential other state and trait factors) interact to impact the altitude training-response in both elite and recreational athletes.

One of these potentially crucial factors that could play a role in the effectiveness of altitude training to trigger performance-improving adaptations is sleep. For example, in the context of acute mountain sickness (AMS), sleep disturbances, and altitude tolerance have already been associated. Nespoulet et al. (2012) compared the altitude-induced sleep-breathing disorders in 12 AMS-susceptible and 12 AMS-non-susceptible individuals and found distinct changes in mean blood oxygen saturation, apnea/hypopnea index (AHI; i.e., the number of significant respiratory events qualifying as apnea or hypopnea per hour of sleep) and hypoxic chemoresponsiveness between both groups of individuals. However, as is known, association is not causation, and distinct kinetics of altitude-induced sleep disturbances and AMS have been demonstrated during a high-altitude sojourn (Nussbaumer-Ochsner et al., 2012). Nussbaumer-Ochsner et al. (2012) reported that, periodic breathing constantly increased over time, while micro arousals and AMS first increased and then decreased over time at altitude. These findings suggest a potential dissociation between periodic breathing and AMS and resulted in the discussion of whether sleep disturbance is a symptom of AMS, or rather an effect of hypoxia *per se* (Roach et al., 2018). Recently, this discussion led to the removal of sleep disturbances from the Lake Louise AMS score to diagnose AMS (Roach et al., 2018). The above emphasizes the importance of interindividual differences in sleep disturbances at altitude and their relative dissociation with AMS.

Specifically within the field of altitude training research, sleep has also already been mentioned (Kinsman et al., 2002, 2005; Hoshikawa et al., 2007; Sargent et al., 2013; Hrozanova et al., 2021; Vitale et al., 2022). Sleep is one of the most important aspects of recovery, and nowadays it is recommended to stay below 3,000 m (or an equivalent normobaric reduction of inspired O_2_) at night in altitude training paradigms (Lundby et al., 2012). This recommendation is based on the fact that sleep is impaired at high altitude (West et al., 2013), and impaired sleep could counteract the positive physiological responses that are aimed for, certainly when it is prolonged for ∼2–3 weeks [i.e., the current suggested optimal hypoxic dose, taking into account altitude and exposure time (Nummela et al., 2021)]. However, the guideline to stay below 3,000 m to prevent altitude-induced sleep impairments might be inadequate. Hoshikawa et al. (2007) demonstrated that acute exposure to normobaric hypoxia equivalent to a 2,000 m altitude decreased slow-wave sleep in athletes, but it did not change subjective sleepiness or amounts of urinary catecholamines. These results point out that the athlete’s sleep might be disturbed even at moderate altitudes of 2,000 m and, more importantly, that athletes are not aware of it (i.e., subjective sleepiness did not change). This is not a novel result: in sleep research, it has been known for decades that sleep-deprivation induced performance decrements are not perceived adequately by participants (e.g., Dongen et al., 2003). Moreover, the AHI increased in hypoxia compared to normoxia, and the magnitude of this effect varied widely among participants (i.e., high interindividual variability) (Hoshikawa et al., 2007).

The current position paper aims to zoom in on a possible role of sleep in intra- and interindividual variability in altitude training-associated responses and to consider altitude training as the medical intervention it actually is. Given the high interindividual variability in the hypoxia-induced increase in AHI (Hoshikawa et al., 2007), the benefits of hypoxia may outweigh any adverse effect of hypoxia on sleep on a group level. However, on an individual level, it might not hold true. Meaning that, for certain individuals, the benefits of exposure to hypoxia may not outweigh the adverse effect of increased arousal and sleep disruption on an athlete’s productivity and recovery. This negative interaction between sleep loss and recovery is well documented in the review of Chennaoui et al. (2015). Both acute and chronic sleep loss are associated with elevated levels of cortisol and inflammation and decreased levels of cortisol and growth hormone (Chennaoui et al., 2015). Effects that may interfere with tissue repair and growth and, eventually, result in overreaching and overtraining, and not attaining the altitude training-response that was aimed for. For example, in patients with obstructive sleep apnea syndrome (i.e., a syndrome that, similarly to hypoxia, results in a significant increase in AHI), the increased AHI creates a noxious environment prone to sympathetic excitation that eventually leads to a chronotropic disability and elevated blood pressure (Stavrou et al., 2021). Moreover, the desaturation that occurs during sleep in these patients (i.e., intermittent hypoxia) results in reduced pulmonary ventilation activity and instability in the ventilatory control system (Stavrou et al., 2021). In the case that, for specific individuals, altitude training has more disadvantages than advantages, altitude training should only be applied following the principle “primum non nocere.” Primum non nocere is a fundamental principle for everyone that is active within the healthcare sector and even beyond, and is applicable to any medical intervention. It means “first, do not harm.” For altitude training, it can be interpreted as “if the risk of causing more harm than good is too big, then the non-application of altitude training may be better than performing it anyway.” As such, this principle links back to the individualized application of altitude training. For further research purposes, we will define the variables to take into account for a full picture of the sleep response to altitude training, whereas, for implementation purposes, we will define how to take sleep into account to individualize altitude training and maximize the training adaptations that are aimed for.

## Sleep at altitude

Barcroft (1920), who spent 6 days in a chamber with lowered oxygen partial pressure to simulate an equivalent altitude of 4,877 m, was the first to report that normobaric hypoxia affected sleep quality (light sleep predominated). Sleep and sleep quality can neurophysiologically be assessed by a technique called polysomnography. Polysomnography refers to the simultaneous measurement of electroencephalography, electrooculography, electromyography, electrocardiography, respiratory movements (chest and abdominal belts) and nasal airflow, and oxyhemoglobin saturation while sleeping. These measurements can eventually be used to categorize sleep in non-rapid eye-movement (NREM) sleep (which can be further subdivided in N1, N2, and N3 stages, from light to deep sleep) and rapid-eye movement (REM) sleep. The distribution of these different sleep stages over the course of one night is a hypnogram, which allows for an objective quantification of sleep architecture, hereby summarizing both sleep quantity and quality. Following the results of Barcroft (1920), further anecdotal evidence of the hypoxia-associated decrease in sleep quality was provided by George I. Finch (Ward, 1993). George I. Finch was a team member of the ill-fated 1924 expedition in which it was attempted to summit Mount Everest (Ward, 1993), and he commented that using supplemental oxygen at night (“sleeping oxygen” was administered at a rate of 1 L.min^–1^) improved sleep (Ward, 1993). This was later confirmed by Pugh, who reported on the scientific aspects of the first successful ascent to Mount Everest (Pugh, 1954). During that ascent, supplemental oxygen improved sleep, provided the perception of warmth and promoted recovery from fatigue (Pugh, 1954). Since these initial anecdotal observations regarding sleep at altitude, many normobaric hypoxic (Rojc et al., 2014; Morrison et al., 2017) and hypobaric hypoxic field (Reite et al., 1975; Szymczak et al., 2009; Johnson et al., 2010; Stadelmann et al., 2013; Fernandez Tellez et al., 2014; Bloch et al., 2015; Pattyn et al., 2017; Bian et al., 2019; Mairesse et al., 2019) and laboratory (Anholm et al., 1992; Houston, 1997; Richalet, 2010) studies focused on the analysis of sleep at altitude, confirming that increasing altitude also increases the level of sleep disturbance.

Overall, sleeping at altitude results in an increased time spent in light sleep (N1 and N2) and a decreased amount of deep sleep (N3, also called slow-wave sleep) (West et al., 2013). With, according to a detailed review of Bloch et al. (2015), the altitude-associated decrease in slow-wave sleep being the most consistent change in sleep that is reported by the few well-designed polysomnographic studies performed in healthy lowlanders arriving at altitude. The impact of altitude on REM sleep has been less straightforward, with some studies reporting a decrease in the amount of REM sleep (Anholm et al., 1992) and others reporting no impact at all (Johnson et al., 2010). Most probably, hard-to-avoid confounding factors such as a new environment (hence a lot of new stimuli to process, thereby increasing REM sleep) and cold ambient temperatures would play a role in the occurrence of these varying results regarding REM sleep. For example, cold ambient temperature is known to decrease the amount of REM sleep and increase the amount of N3 (Buguet et al., 1998). Besides specific sleep stages, altitude also affects the number of arousals and the breathing pattern during sleep (West et al., 2013). An altitude-associated increase in the number of arousals has been consistently reported in multiple studies (Reite et al., 1975; Salvaggio et al., 1998; Zieliński et al., 2000; Van Cutsem et al., 2022), and might very well be the key variable in altitude-induced changes in sleep architecture. Periodic breathing can be defined as an oscillatory behavior with alternating periods of hyperventilation followed by central apneas or hypopneas (Bloch et al., 2010) and is thought to, in part, underly the hypoxia-associated deteriorations in sleep architecture and increase in arousals (West et al., 2013; Van Cutsem et al., 2022). Moreover, in contrast to some other hypoxia-induced changes during sleep [e.g., blood oxygen saturation levels (Bloch et al., 2010; Nussbaumer-Ochsner et al., 2012)], periodic breathing seems to persist over time at altitude and does not partially restore after a couple of acclimatization days (Bloch et al., 2010; Fernandez Tellez et al., 2014). Bloch et al. (2010) studied nocturnal breathing patterns in 34 mountaineers and observed a persistence of periodic breathing over a several-week period. In addition, Fernandez Tellez et al. (2014) conducted a study at an Antarctic research station “Concordia.” Concordia is located at 3,200 m above sea level, but based on barometric pressure, the inspired O_2_ is an equivalent of approximately 3,800 m. Fernandez Tellez et al. (2014) included 13 Antarctic overwinterers and found that during the entire 13-month campaign, the periodic breathing response remained stable for all participants, whether they showed a high or a low vulnerability to it. Again, this result suggests a strong trait-like component in this effect. Importantly, periodic breathing typically occurs during NREM sleep and not during REM sleep (West et al., 2013). Within NREM sleep, N3 is known to be the physiologically restorative sleep phase (Taylor et al., 1997; Halson and Juliff, 2017). It plays an important role in, for example, the secretion of growth hormone (Van Cauter and Plat, 1996). As such, it would be a crucial phase in a healthy compensation response in any physically challenging situation, like training for an elite athlete, and most definitely altitude training. Any physiological mechanism relying on cellular growth requires an optimal growth hormone secretion. In addition, periodic breathing and specifically the associated sleep apneas and hypopneas also result in a repetitive aggravation of the altitude-induced desaturation throughout the sleep period. This intermittent desaturation, as also encountered in obstructive sleep apnea syndrome patients, is well known to have specific physiopathological consequences on the overall health status, with systemic effects such as oxidative stress, inflammation, and cardiovascular or metabolic impairments, that may be particularly deleterious for an athlete’s training response and performance (Stavrou et al., 2021).

As such, the presence of altitude-associated periodic breathing appears to be an important phenomenon to consider when measuring the effectiveness of an altitude training protocol. Athletes experiencing disturbed/impaired sleep due to periodic breathing will reduce their productivity and impair recovery (Aguillard et al., 1998). In addition, this decrease in productivity and impaired recovery may or may not [see the results of Hoshikawa et al. (2007)] be consciously perceived as somnolence and/or fatigue. If consciously perceived, the combination of the objective and subjective effects of nocturnal periodic breathing could further impair productivity and recovery. In the review of Chennaoui et al. (2015) the different physiological and psychological pathways through which sleep and physical activity impact each other have been well described. Acute sleep loss has been observed to result in immune-inflammatory changes such as increased pro-inflammatory cytokine, growth hormone and testosterone concentrations after physical exercise (Abedelmalek et al., 2013) and to down regulate activity of the protein synthesis pathway that repairs muscle damage and trigger contractile function deficits during recovery (Dattilo et al., 2011). While in terms of chronic sleep restriction, Haack et al. (2007) reported that reducing sleep duration to 4 h/night across 10 days increased levels of plasma interleukin-6 and increased pain ratings. In addition, Leeuwen et al. (2010) found that spending 4 h/night in bed for 5 days increased insulin and leptin levels as well as the insulin-to-glucose ratio. In light of the present paper, the most important aspect of the interaction between sleep and exercise is the fact that both acute and chronic sleep loss are associated with elevated levels of cortisol and inflammation and decreased levels of cortisol and growth hormone (Chennaoui et al., 2015). Effects that may interfere with tissue repair and growth and, eventually, result in overreaching and overtraining, and not attaining the altitude training-response that was aimed for. Given the high occurrence of altitude-associated sleep impairments (see the sections above and below), and the important role of slow-wave sleep in avoiding overreaching/overtraining during periods of high volume training (e.g., during an altitude training camp), it would be unethical not to consider these risks when planning an altitude training camp with athletes.

Eventually, it’s clear that altitude-associated periodic breathing and the associated sleep impairments can reduce the effectiveness of the altitude training protocol to increase an athlete’s sea-level performance. Therefore, to eventually be able to positively impact sleep at altitude, it is important to gain insight in the physiology underlying altitude-associated periodic breathing (i.e., the main mediating factor of the negative impact of altitude on sleep). To do so, a basic understanding of the ventilatory control system during sleep at altitude is necessary.

### Ventilatory control during sleep at altitude

Unlike the heart, which has its own rhythmic control and muscle activity within one organ (albeit under influence of several nervous pathways), breathing requires the interplay of a brain control center and a peripheral muscle effector system. The ventilatory control system consists of three main components (see Figure 1): (1) the respiratory centers in the central nervous system, which are responsible for the genesis of the respiratory drive; (2) the effector system, i.e., the ventilatory muscles of the thorax and neck; and (3) the receptors (mechanoreceptors in the lungs, and peripheral and central chemoreceptors sensitive to blood gases and pH), which inform the respiratory control centers of necessary adaptation to the ventilatory drive (Hermand et al., 2015). This system is a closed loop which, in usual circumstances, produces a relatively stable level of ventilation (Hermand et al., 2015). However, in some cases, the system shows a marked degree of instability that eventually can result in periodic breathing. Hypoxia is such a “case” in which instability is triggered (Hermand et al., 2015). More specifically, this instability results from a time delay of the O_2_/CO_2_ feedback that is generated by the chemoreceptors (i.e., central and peripheral) to the respiratory centers (Hermand et al., 2015). This time delay is linked to the lung-to-chemoreceptors circulation time, i.e., it takes some time for blood gases (O_2_ and CO_2_) to transit from the lungs to the chemoreceptors, and therefore it takes some time for changes in arterial O_2_ and CO_2_ concentrations to be detected by chemoreceptors. Simply put, exposure to hypoxia will lead to a drop in partial pressure of arterial O_2_ (PaO_2_) and acid-base adjustments, ensued by alterations in chemoreflex control and cerebrovascular responses to changes in arterial blood gases (i.e., PaO_2_ and PaCO_2_). The alterations in the chemoreflex control (i.e., increased ventilatory sensitivity) during hypoxia causes the feedback system to overshoot and to trigger hyperventilation. This hyperventilation will eventually result in hypocapnia (i.e., a drop in PaCO_2_) and thus, an increase in pH (respiratory alkalosis). Hypocapnia and alkalosis are sensed by chemoreceptors that signal back to the respiratory centers to suppress the respiratory output, possibly leading to an apnea, which provides an opportunity for PaCO_2_ to rise again (see Figure 1 for an overview) (Ainslie et al., 2013; Kong, 2021). Particularly during sleep, when ventilation is lower and resting PaCO_2_ is higher compared to awake (i.e., the delta between resting PaCO_2_ and the PaCO_2_-apnea threshold is small), the hypoxia-related increase in chemoreflex sensitivity and eventual over-hyperventilation will most easily introduce instability in the ventilatory control system and result in periodic breathing (Ainslie and Duffin, 2009; Ainslie et al., 2013). For a more detailed description on the mechanisms underlying periodic breathing, we refer to Ainslie and Duffin (2009) and Ainslie et al. (2013) and particularly Figure 13 in Ainslie and Duffin (2009) and Figure 12 in Ainslie et al. (2013). For an example on how the time delay in O_2_/CO_2_ feedback eventually can result in an oscillatory ventilation pattern (i.e., periodic breathing) at altitude, see West et al. (2013).

**FIGURE 1:** Graphical overview of the ventilatory control system and the hypoxia-associated cascade (i.e., step 1–8) that eventually could trigger periodic breathing during sleep.

### Sleep at altitude during altitude training protocols

We have described in Section “Sleep at altitude” how sleep is impaired at altitude, and how these impairments could be critical for athletes. In the present section, we will further zoom in on existing sleep research that has been performed within the field of altitude training (Kinsman et al., 2002, 2005; Hoshikawa et al., 2007; Sargent et al., 2013; Hrozanova et al., 2021; Vitale et al., 2022). We have only reviewed literature reporting polysomnography, as sleep architecture in altitude settings can only accurately be described by this methodological gold standard (e.g., Pattyn et al., 2018).

Kinsman et al. (2002) were the first to monitor polysomnography in athletes undertaking a LHTL protocol. They set out to evaluate the acute effects of sleeping at a simulated moderate altitude of 2,650 m (Kinsman et al., 2002) and hypothesized that LHTL athletes may exhibit some respiratory events during sleep, but that periodic breathing, *per se*, would not occur under moderate hypoxia. This hypothesis was based on the fact that 2,650 m was well below the minimum at which periodic breathing during sleep had been observed back then, and on research suggesting an association between intensive exercise training (i.e., elite athletes) and a depressed hypoxic ventilatory response (HVR; i.e., a measure of ventilatory sensitivity; see Sections “Intra- and inter-individual variability in altitude-associated sleep impairments” and “Genetic markers associated with altitude-associated sleep impairments” for more information) (Kinsman et al., 2002). According to this hypothesis, the depressed HVR would lead to a more stable ventilatory control system in athletes. Nevertheless, their study established that nocturnal normobaric hypoxia simulating an altitude of 2,650 m has acute effects on breathing during sleep of most athletes and that the magnitude of these effects varies widely between individuals (Kinsman et al., 2002). Moreover, periodic breathing occurred in nearly 25% of their participants (i.e., 4 out of 17) (Kinsman et al., 2002). Following up on this first study, Kinsman et al. (2005) performed a second study, in which they monitored sleep throughout a 15-day LHTL protocol, to investigate beyond acute effects. This follow-up study showed significant increases in arousal and respiratory disturbance indices on nights 8 and 15 of simulated altitude (i.e., 2,650 m) versus baseline near sea level (Kinsman et al., 2005). NREM sleep was unchanged over time, while REM sleep increased on night 8 and 15 compared to night 1 of simulated altitude (Kinsman et al., 2005). The authors concluded that the increase in REM sleep over time might be indicative of acclimation, but that it is unsure whether this acclimation-associated change in sleep architecture balances any physiological detriment caused by more arousals and increased respiratory disturbance index over the 15 nights (i.e., no acclimation-associated change occurred in these specific measures). Regarding this lack of acclimation-associated changes in respiratory disturbance indices and arousals, Kinsman et al. (2005) put forward that “*it is conceivable that in the case of athletes using nightly hypoxia in an attempt to gain a small performance advantage, the benefits of nocturnal exposure may outweigh any adverse effect of increased arousal and sleep disruption.”*. Given the high interindividual variability, that was emphasized again in the second study of Kinsman et al. (2005), this statement might hold true on a group level, it might, however, not hold true on an individual level. Meaning that, for certain individuals, the benefits of nocturnal exposure to hypoxia may not outweigh the adverse effect of increased arousal and sleep disruption.

The study of Kinsman et al. (2002) and Kinsman et al. (2005) demonstrated that nocturnal periodic breathing occurred acutely in athletes when residing at a simulated moderate altitude of 2,650 m, and, more importantly, also showed that this negative effect of altitude on sleep-disordered breathing did not dissipate throughout a 15-day LHTL protocol. These investigations were followed up by multiple other research teams (Hoshikawa et al., 2007; Sargent et al., 2013; Hrozanova et al., 2021; Vitale et al., 2022). However, only two of them also used polysomnography (i.e., the gold standard) to evaluate sleep (Hoshikawa et al., 2007; Sargent et al., 2013). Without polysomnography, the interpretation of sleep is restricted to a proxy measure of sleep quantity, and no interpretation of sleep architecture (Conley et al., 2019). Polysomnography measures the neurophysiological process of sleep. Actigraphy (the basic mechanism of all other proxy measurements) measures a behavior (movement). Hoshikawa et al. (2007) revealed that acute exposure to normobaric hypoxia, even at an equivalent of 2,000 m altitude, negatively impacts sleep. Sargent et al. (2013) showed the lack of acclimatization-associated changes in periodic breathing during a 2-week altitude training camp in La Paz (3,600 m) in 10 under-17 elite soccer players. In addition, Sargent et al. (2013) found that REM sleep did return to normal after 2 weeks at altitude. The results of Hoshikawa et al. (2007) and Sargent et al. (2013) further substantiate the results of Kinsman et al. (2005) and confirm that some aspects of sleep seem to improve with prolonged exposure to altitude (i.e., REM sleep), while others do not at all (i.e., periodic breathing).

The role of sleep in altitude training was also shortly mentioned in the critical review of Lundby et al. (2012). Based on the study of Nussbaumer-Ochsner et al. (2012), they suggested that sleep quality is rapidly increased with acclimatization to altitude (i.e., within three nights) and, as such, implicitly question any role of importance for sleep in intra- and interindividual variability in the altitude training-associated responses (Lundby et al., 2012). The data of Nussbaumer-Ochsner et al. (2012) demonstrates that sleep does improve with acclimatization to altitude, however, not to an extent that sleep quality is restored to sea level-values. For example, it was demonstrated that, after three nights at altitude (4,559 m), median nocturnal oxygen saturation improved from 67% during night 1 to 71% (sea level-value was 96%), the amount of relative slow wave sleep improved from 6% during night 1 to 11% (sea level-value was 18%) and the AHI didn’t improve at all and was 60.9/h during night 1 and 86.5/h during night 3 (sea level-value was 0.1/h) (Nussbaumer-Ochsner et al., 2012). Subsequently, rather than demonstrating that acclimatization to altitude rapidly restores/improves sleep quality and periodic breathing, the data of Nussbaumer-Ochsner et al. (2012) reconfirms the findings of the above mentioned sleep research within the altitude training-research field, i.e., acclimatization to altitude does not restore/improve altitude-associated periodic breathing throughout the length of a typical altitude training protocol. Again, this is further demonstrated by specific sleep research, like the results from Bloch et al. (2010) or Fernandez Tellez et al. (2014), which we already discussed.

Based on the above, it seems fair to say that sleep, and more specifically the prolonged negative impact of altitude on the nocturnal breathing pattern, and hence on the amount of deep sleep, could play an important role in intra- and interindividual variability in the altitude training-associated responses in athletes.

## The role of physical activity in altitude-associated sleep impairments

The previous sections point out how the negative impact of hypoxia on the ventilatory control system appears to be one of the main mediators of impaired sleep at altitude, and summarized that this impact of hypoxia on sleep also occurs in athletes throughout an altitude training camp. However, while completing an altitude training camp, hypoxia is not the only physiological stressor known to have an impact on the ventilatory control system. Intense physical activity is another variable and, considering the logical high amount of physical load that is incorporated in every altitude training protocol, a very important one. In addition to hypoxia, the combination of exercise and hypoxia may acutely introduce even more instability in the ventilatory control system. Because, even in hypoxic conditions, exercise by itself induces a further drop in PaO_2_ and arterial oxygen saturation (Woorons et al., 2007; Hermand et al., 2015). PaO_2_ dropping further could result in an even higher increase in ventilatory sensitivity, which subsequently could lead to a greater over-hyperventilation and destabilization of the ventilatory control system (see Figure 1).

The acute effect of exercise on the HVR (i.e., a measure of ventilatory sensitivity) has been long studied. Weil et al. (1972) already reported a marked increase in the HVR during mild exercise. Recently, Yamashiro et al. (2021) reconfirmed that both peripheral and central chemosensitivity to CO_2_ increases during mild exercise, with the peripheral chemoreceptors playing a dominant role. Moreover, they also demonstrated that, when combined with exercise, the effect of CO_2_ inhalation on ventilation is not additive to the effect of exercise on ventilation, but is significantly larger and thus appears to be interactive (Yamashiro et al., 2021) [see Figure 4 in the publication of Yamashiro et al. (2021)]. In addition, Constantini et al. (2021) also reported that ventilatory responsiveness to progressive hypoxia is augmented during exercise. Based on the above, the acute effect of exercise and hypoxia on the ventilatory control system appears to interact, leading to an even greater impact on the system.

Besides this acute interaction, exercise and hypoxia might also reinforce each other’s impact on the ventilatory control system at the subacute/chronic level. Levine et al. (1992) evaluated the HVR before and after 5 weeks of cycle ergometer training at either sea level or 2,500 m in 21 untrained men and women. Their results showed that 5 weeks of endurance training at sea level has no effect on the HVR. However, when endurance training is performed at altitude, the HVR is increased (Levine et al., 1992). Unfortunately, Levine et al. (1992) did not design their study to statistically evaluate a possible interaction effect between exercise training and hypoxia, for example, by including a condition in which individuals were exposed to 5 weeks of intermittent altitude exposure without exercise training. As such, the increase in the HVR after 5 weeks of cycle ergometer training at 2,500 m could also be interpreted as a normal acclimatization-associated process, independent of the exercise training. Nevertheless, Levine et al. (1992) do provide some compelling arguments [e.g., during the 5 weeks of endurance training participants were only exposed to hypoxia during the exercise training (i.e., intermittent altitude exposure)] to substantiate their interpretation that the metabolic and/or hemodynamic stimulus of exercise, in combination with hypoxia interact to cause a sustained increase in chemosensitivity, that is manifested as an increase in the HVR (Levine et al., 1992). The exact nature of the hypoxia-exercise interaction could, however, not be further elucidated by the study of Levine et al. (1992) and, up to date, the evidence on an interaction between exercise training and altitude exposure on ventilatory control is still scarce. Nonetheless, data suggesting a possible interaction between exercise training and altitude exposure can also be found in some other research areas. For example, Tellez et al. (2016) ran two experiments, one in confined, normobaric hypoxic conditions (i.e., a 10-day study at an altitude equivalent to 4,000 m) in a laboratory situation, and another one in confined, hypobaric hypoxic conditions at the Concordia Antarctic Research Station (i.e., a 13-month study at an altitude of 3,800 m), and established that performing physical activity can exacerbate the number of hypoxia-induced nocturnal apneas and hypopneas. Tellez et al. (2016) suggested that the exercise-evoked sympathetic activation increases chemoreceptor sensitivity and subsequently also further increases the occurrence of periodic breathing at altitude. The exercise-evoked sympathetic activation that is hypothesized to further increase the occurrence of periodic breathing at altitude can persist up to 6 days after an exercise session is completed (Eyzaguirre and Lewin, 1961). During the nights following on the exercise session, the negative interaction effect of physical activity and hypoxia might thus persist, and further decrease the quality of physical recovery.

The possible interaction between hypoxia and exercise goes to show that performing physical activity at altitude or, in case of executing a LHTL protocol, right before going to altitude, might exacerbate nocturnal periodic breathing, and that the interaction between physical activity and altitude needs to be considered to optimize altitude training protocols in both elite and recreational athletes. However, further research is necessary to substantiate that the effects of hypoxia and physical activity on the ventilatory control system interact and, subsequently, to elucidate the precise physiological mechanism underlying this interaction.

## Intra- and interindividual variability in altitude-associated sleep impairments

Similarly to the effectiveness of altitude training to improve athletic performance, significant intra- and interindividual differences are present in the altitude-associated sleep impairments (Fernandez Tellez et al., 2014). However, unlike the interindividual differences in the altitude training-associated responses, Fernandez Tellez et al. (2014) demonstrated that the interindividual differences in the altitude-induced changes in the AHI and nocturnal arterial O_2_ saturation remained stable over time (i.e., over a period as long as 13 months). Moreover, the interindividual differences in the altitude-induced changes in the AHI were found to be substantive (Fernandez Tellez et al., 2014). The fact that these interindividual differences appear to be stable in time indicates that, unlike for the responsiveness to altitude training, altitude-induced changes in sleep can be classified as a trait. This provides an opportunity to elucidate the factors that determine the presence of this trait for any given individual and hence, to be able to detect individuals that are predisposed to experience impaired ventilatory control and sleep at altitude.

A factor that has been focused on in the quest for the underlying mediators of the intra- and interindividual variability in altitude-associated sleep impairments is endurance training. The first sleep study within the research field of altitude training hypothesized that athletes may be less susceptible to altitude-induced respiratory disturbances, due to exercise training being associated with a depressed HVR (Kinsman et al., 2002). As such, Kinsman et al. (2002) put forward exercise training as an important factor to explain part of the interindividual variability that is present in altitude-induced respiratory disturbances. To back up this hypothesis, Kinsman et al. (2002) referred to, amongst others, the study of Byrne-Quinn et al. (1971). Byrne-Quinn et al. (1971) demonstrated that athletes, compared with non-athletes, have a decreased hypoxic ventilatory drive at rest (Byrne-Quinn et al., 1971). Subsequently, this observation led to the extrapolation that the peripheral chemoreceptor function in athletes is decreased, and that exercise training might make individuals less susceptible to altitude-induced respiratory disturbances. However, the results of Kinsman et al. (2002) eventually pointed out that a LHTL protocol at moderate simulated altitude can cause substantial respiratory events during elite athlete’s sleep. As such, regular exercise training does not seem to fully counteract altitude-induced respiratory disturbances and sleep impairments at altitude can be expected in all populations: elite, recreational and sedentary individuals. Nonetheless, these results do not exclude that being endurance trained might still explain some part of the interindividual differences in altitude-induced respiratory disturbances and provide some buffering to it. The study of Kinsman et al. (2002) does, however, not provide any additional insight on this matter, as it was not designed for this purpose (i.e., there was no matched sedentary group included). Levine et al. (1992) specifically focused on a role for endurance training in the differing HVR between athletes and non-athletes (i.e., the role of endurance training in interindividual differences in altitude-associated respiratory disturbances). These authors evaluated the longitudinal effect of 5 weeks of endurance training on the HVR, and concluded that endurance training at sea level had no effect on the HVR, suggesting that the role of physical training in a blunted HVR and hence resilience to altitude-induced respiratory disturbances is rather limited. Despite the fact that it cannot be excluded that a more prolonged duration of endurance training, over months or years, might be sufficient to result in a blunted HVR, their findings indicate that genetic or other environmental factors may be more important in determining a depressed hypoxic drive in endurance athletes compared to non-athletes (Levine et al., 1992).

Within a sporting context, the factors underlying the depressed HVR in athletes compared to non-athletes are relevant. However, even more relevant, are the factors underlying the intra- and interindividual differences in altitude-induced respiratory disturbances within an elite athlete population itself. Kinsman et al. (2002) hypothesized that a decreased HVR could lead to less periodic breathing at altitude and therefore facilitate altitude training-associated physiological changes in athletes. However unfortunately, Kinsman et al. (2002) were unable to measure the HVR of their participants because of a technical limitation. Luckily, this hypothesis was also investigated by other research groups that did manage to assess the HVR (Ainslie et al., 2013). Some of this research has been summarized by Ainslie et al. (2013), who concluded that, within a lowlander population, the relationship between the HVR and periodic breathing is complex and sometimes even absent. Nevertheless, these authors also pointed out that, based on the known blunted HVR and diminished periodic breathing in Sherpas, a role of the HVR in periodic breathing is apparent. More specifically, regarding a sporting context, the added value of the HVR in determining individuals who might be more susceptible to develop periodic breathing at altitude has also been emphasized by Chapman (2013). Based on anecdotal evidence, he reported that the few athletes who demonstrate relatively strong HVRs (i.e., greater than ∼0.5 L/min/% arterial oxygen saturation) typically demonstrate the most dyspnea and perceived exertion during training on arrival and throughout training at moderate altitude (Chapman, 2013). Subsequently, Chapman (2013) also put forward that these athletes tend to struggle more with workouts and may be better off staying at sea level to train. In contrast, Turner et al. (2022) recently published data that demonstrates that, in a group of 14 elite endurance runners who completed a 4-weeks LHTH (∼2,400 m) camp, an elevated HVR at rest was associated with an enhanced total hemoglobin mass after the LHTH training camp. However, important to note is that, based on a visual interpretation of Figure 2B in the paper of Turner et al. (2022), all elite runners had a relative HVR (body weight is taken into account) around or below the threshold that was put forward by Chapman (2013) (i.e., ∼0.5 L/min/% arterial oxygen saturation). Certainly when this threshold is also made relative to body weight. For example, for an individual of 70 kg the relative threshold would be ∼0.7 L/min/% arterial oxygen saturation/kg. As such, it appears that, below a certain threshold, an elevated HVR at rest could be beneficial to enhance the altitude training-associated increase in total hemoglobin mass and thus not result in respiratory disturbances that impair altitude training-induced responses.

The above substantiates that interindividual differences in the HVR and the associated altitude-induced respiratory disturbances contain valuable information and, as already suggested by Turner et al. (2022), could provide an opportunity to coaches and practitioners to optimize and individualize acclimatization strategies and altitude training methods. However, it is clear that, the relation between the HVR at rest, altitude-induced respiratory disturbances (e.g., periodic breathing) and altitude training-associated physiological changes (e.g., an increase in total hemoglobin mass) will certainly not be linear, but rather complex. Moreover, endurance training appears to explain only a limited part of the interindividual variability that is present in the HVR and the altitude-associated respiratory disturbances. As such, other factors [e.g., genetic or other environmental factors (Levine et al., 1992)] that result in this interindividual variability should be elucidated. A candidate proxy to play a role in the ventilatory response to hypoxia is genetics (Weil, 2003).

### Genetic markers associated with altitude-associated sleep impairments

Weil (2003) was the first to summarize the available evidence from family and population studies which shows a genetic influence in the ventilatory response to hypoxia. They concluded that ventilatory responses to hypoxia vary among human subjects within familial clusters, which together with concordance among identical twins definitely points toward a strong hereditary component (Weil, 2003). However, at the time, no clear clues to the identity of the relevant genes could be put forward (Weil, 2003). Up to date, research by both Goldberg et al. (2017) and Lancaster et al. (2020) followed up on the study of Weil (2003), and provides insight into the genes determining the HVR. Goldberg et al. (2017) evaluated the association between the hypoxic and hypercapnic ventilatory response on the one hand, and coding variants in genes participating in breathing on the other hand (i.e., the PHOX2B, GPR4, and TASK2/KCNK5 gene) in 551 healthy young adults. They found that two TASK2/KCNK5 variants (rs2815118 and rs150380866) played a role in the hypercapnic ventilatory response (Goldberg et al., 2017). In addition, Goldberg et al. (2017) also demonstrated a sex difference in the HVR. The HVR of men is 31,2% higher compared to women, and although there is conflicting evidence (see Goldberg et al., 2017 for a discussion), the data of Goldberg et al. (2017) indicate that men could be more susceptible to develop altitude-associated periodic breathing. The study of Lancaster et al. (2020) assessed the role of selective antioxidative (SOD2, CAT, and GPX) and neurodevelopmental (NOTCH4 and BDNF) genes in specific features of periodic breathing in 22 healthy subjects. Polymorphisms in the NOTCH4 (rs367398) and CAT (rs1001179) genes were demonstrated to impact periodic breathing incidence during hypoxia (Lancaster et al., 2020). In case of the rs367398 polymorphism in the NOTCH4 gene, the presence of an A allele was found to result in more pronounced periodic breathing (Lancaster et al., 2020). Whereas, for the rs1001179 polymorphism in the CAT gene, the presence of a T allele resulted in less pronounced periodic breathing (Lancaster et al., 2020). However, before being able to pinpoint individuals that are genetically more susceptible to develop periodic breathing at altitude, these exploratory findings need further replication in future studies with large sample sizes, and more importantly taking into account all the potential moderating variables of the combined hypoxia-exercise response. Indeed, it is clear that in order to determine the periodic breathing-susceptibility of an individual, other factors besides genetic set-up will have to be taken into account (Narang et al., 2022). For example, Narang et al. (2022) put forward that a blunted resting, but not exercising, HVR has been observed in pre-term adults, and subsequently speculated that pre-term birth could protect against the consequences of exercise combined with hypoxia.

## How to improve altitude training-effectiveness by taking sleep into account

In the first paragraph of the current paper, we already referred to the study of Nummela et al. (2021). These authors demonstrated that considering factors known to underly intra- and interindividual variability in the effectiveness of altitude training is worthwhile (Nummela et al., 2021). Our review of the literature within both sleep and altitude training fields points out that, besides altitude, iron deficiency, and inflammation, sleep is another factor that could impact the effectiveness of altitude training protocols. To optimize the altitude training-response, Nummela et al. (2021) determined an optimal altitude dose (2,000–2,500 m), a low cut-off for iron deficiency (pre-S-Ferritin > 30 μg/L) and a high cut-off for inflammation (pre-S-hs-CRP < 3 mg/L). To further increase the effectiveness of altitude training by taking sleep into account, interventions that positively impact altitude-associated periodic breathing (i.e., the main mediator of the altitude-associated decrease in deep sleep, and the interaction nexus between physical activity and altitude) need to be developed. Subsequently, the individualized application of these interventions should improve physical recovery during sleep and, as such, the effectiveness of altitude training (see Section “Altitude-associated periodic breathing countermeasures”). To successfully individualize countermeasures, individuals who are predisposed to altitude-associated sleep impairments need to be determined, which we further discuss in one of the following paragraphs. The determination of this trait-like predisposition should, together with state variables such as iron deficiency and inflammation, eventually be included in the decision process that aims to conclude whether the benefits of altitude training will outweigh the disadvantages for a given athlete.

### Altitude-associated periodic breathing countermeasures

Building on the growing understanding of the mechanisms underlying periodic breathing at altitude, multiple interventions have been developed and investigated. In general, the currently available periodic breathing-countermeasures can be subdivided in a pharmacological and a non-pharmacological category. Pharmacologically, products such as acetazolamide, dexamethasone, various hypnotics and theophylline have been evaluated and found to be effective to a certain degree (Ainslie et al., 2013). However, within a sporting context, most of these products are inapplicable, due to being part of the World Anti-Doping Agency Prohibited list (e.g., acetazolamide). Within the non-pharmacological category, an additional subdivision can be made by distinguishing between devices and nutritional countermeasures. In terms of devices, bi-level positive airway and the addition of dead space *via* a modified facemask have been shown to positively impact certain aspects of sleep at altitude (Ainslie et al., 2013). Regarding nutrition interventions, Patrician et al. (2018) were unable to improve the nocturnal breathing pattern or oxygenation with dietary nitrate supplementation (i.e., beetroot juice), but did demonstrate that the intake of beetroot juice increased the fluctuations in arterial O_2_ saturation during sleep at altitude. However, similarly to the field of the pharmacological and device-related countermeasures, further research is needed in the field of nutritional countermeasures as well. Both Ainslie et al. (2013) and Kong (2021) provide a complete overview of these countermeasures. One might wonder whether the need to alleviate the nocturnal hypoxia associated with sleeping at altitude during altitude training protocols does not mean the athlete would be better off sleeping at sea level. Nocturnal hypoxia countermeasures are relevant in contexts like mountain expeditions. However, in the context of altitude training protocols, if a specific athlete seems to be exposed to more risks due to impaired sleep than benefits due to nocturnal hypoxia exposure, the obvious solution would be to keep him/her sleeping at sea level.

### How to determine a predisposition for altitude-associated periodic breathing?

To predict whether someone is predisposed, genetics do appear to be a valid option. However, as we previously discussed (see Section “Genetic markers associated with altitude-associated sleep impairment”), before being able to genetically pinpoint individuals that are more susceptible to develop periodic breathing at altitude further research steps need to be taken. In addition, a hypoxic sensitivity pre-screening that includes the assessment of ventilatory and cardiac responses to hypoxia at rest seems to predict altitude training-associated physiological changes (Turner et al., 2022). However, as with genetic screening, more research is needed before this method of pre-screening can be recommended to assess predisposition to altitude-related periodic breathing and sleep disturbances.

Besides predicting susceptibility to altitude-associated periodic breathing, the monitoring of it can also provide insight in an individuals’ sleep at altitude and lead to the application and individualization of useful countermeasures. To monitor sleep in the field, both objective and subjective tools have been developed (Vlahoyiannis et al., 2020). Objective sleep assessment methods that can be applied in an athlete setting can be subdivided in polysomnography, actigraphy (i.e., a monitoring device that estimates sleep/wake behavior based on accelerometery) and wearables/nearables, applications and consumer technologies (i.e., devices that function in a similar way than actigraphs, but that are typically connected with a remote application). Typical subjective sleep assessment methods are sleep diaries and questionnaires that provide a self-rated estimate of sleep-related parameters [see the review of Vlahoyiannis et al. (2020) for a full overview]. Each one of these sleep assessment methods comes with its pros and cons, and of course the combination of multiple methods can provide a valuable, more holistic insight in a complex phenomenon such as sleep. To choose the most effective combination of sleep assessment methods it is important to know the advantages and disadvantages of each one. First of all, it should be clear that sleep architecture (i.e., the division of a night’s sleep into different sleep stages) can only be attained by making use of polysomnography (Conley et al., 2019; Vlahoyiannis et al., 2020; Miller et al., 2022). Hence, the impact of altitude and exercise on the physiological recovery function of sleep (i.e., the amount of deep sleep), can only be measured through polysomnography. Despite the numerous commercial applications claiming to deliver this outcome, none of them has been reliably and repeatedly validated by independent scientific investigation, which is reflected in the recommendations of all professional sleep medicine societies. Obviously, due to the necessary monitoring of multiple physiological systems, the application of polysomnography in a sport field setting is less straightforward and is often complex. Compared to polysomnography, actigraphy, wearables, sleep diaries, and questionnaires have the advantage that they are less invasive, less costly and require less expertise to be applied and interpreted [see Figure 2 in the review of Vlahoyiannis et al. (2020)]. In terms of subjective sleep assessment methods, as we previously pointed out, the subjective evaluation of sleep does not always reflect sleep disturbances that are objectively noticeable. For example, Hoshikawa et al. (2007) demonstrated that acute exposure to normobaric hypoxia (i.e., equivalent to 2,000 m) decreased slow-wave sleep in athletes, but it did not change subjective sleepiness. Moreover, hypoxia itself is also known to impact the psychological state (Tobita et al., 2022). These results are crucial to keep in mind, because they demonstrate unequivocally that the one alteration of sleep architecture that has potentially the largest impact on physiological recovery might not even be noticed by the athletes who experience it. A combination of objective and subjective sleep assessment methods, with a screening polysomnography allowing to determine sleep architecture and hypoxia responses, seems warranted to detect all sleep impairments. Despite its more complex application in the field, polysomnography should be the first choice to evaluate an individual’s predisposition to altitude-associated sleep impairments. To counteract the major disadvantage of polysomnography (i.e., the complex application in the field and a necessary sleep expert to interpret the gathered data), future research should assess whether the polysomnographic evaluation of one night of sleep at altitude (e.g., in a hypoxic chamber) preceding performing an altitude training protocol is able to detect those individuals whose sleep will most heavily be affected due to altitude during the altitude training camp itself. If this is the case, then a sleep at altitude-evaluation could become a standard evaluation in assessing whether the benefits of altitude training would outweigh the disadvantages for a given individual. If the polysomnographic evaluation of one night of sleep is unable to pinpoint susceptibility to altitude-associated sleep impairments, or if the inclusion of a polysomnographic evaluation of one night of sleep at simulated altitude does not seem reasonable from the athlete and/or staff point of view (e.g., still too time-consuming). Then sleep wearables that specifically aim to monitor sleep related breathing [e.g., the Sunrise device that has been developed to be applied on the chin (Pépin et al., 2020)] or consequences of nocturnal periodic breathing (e.g., the assessment of the nocturnal hypoxic load with nocturnal oximetry could be an easy method to monitor nocturnal intermittent hypoxia) could be the next best option to apply in an athletic population and follow-up sleep and/or periodic breathing throughout an altitude training camp. Independently from whether a polysomnographic evaluation can be included in a sporting context, the development of alternative and easy-to-apply strategies to monitor altitude-associated periodic breathing and its impact on sleep is clearly required.

### Practical recommendations

All the above can be boiled down to the following practical recommendations. (1) *Inform and educate.* Given the possible high impact of sleep impairments on an athlete’s functioning and recovery it is only ethical to inform and educate athletes about the possible impact of altitude training on their sleep. (2) *Screen and monitor.* Besides informing and educating, athletes should be screened for their vulnerability to altitude-associated periodic breathing and related sleep impairments. Such a vulnerability screening should be performed with polysomnography, as sleep architecture in altitude settings can only accurately be described by this methodological gold standard (e.g., Pattyn et al., 2018). In addition to screening, real-time monitoring of the impact of altitude on an athlete’s sleep is also crucial. From a feasibility point of view, both for the athlete and the staff, alternative strategies to polysomnography should be considered to monitor sleep and periodic breathing during altitude training (e.g., nocturnal oximetry). (3) *Consider the pros and cons*. If an athlete’s vulnerability is low to moderate, the pros of performing altitude training may outweigh the cons. In this case, to double check the result of the polysomnographic screening, sleep wearables that have been developed to specifically detect sleep related breathing (e.g., Sunrise) are warranted to follow-up the nocturnal breathing pattern throughout an altitude training camp. If an athlete’s vulnerability is high, the cons may outweigh the pros, and the obvious solution for the athlete would be to refrain from altitude training. Of course, altitude training camps are about more than solely pursuing hypoxia-induced hematological and non-hematological physiological adaptations, e.g., creating cohesion in a group of athletes, isolating an athlete or a group of athletes and create full focus on specific training goals. As such, it is possible that highly vulnerable athletes, still want to participate in an altitude training camp (i.e., when to not lose contact with the team). In addition, throughout a competitive season, athletes could certainly encounter situations in which they have to perform and live at altitude for multiple days (e.g., a cyclist competing in the Tour de France, a judoka participating in a competition that is held in Mexico City). In these cases, i.e., a highly vulnerable athlete is exposed to altitude, hypoxia severity at night should be reduced (e.g., within LHTL settings when individual hypoxic bedrooms are used). Or, if it is impossible to reduce hypoxia severity, periodic-breathing countermeasures should be applied. Within a sporting context, the most promising interventions are the non-pharmacological ones (e.g., the addition of dead space *via* a modified facemask) since many of the pharmacological ones (e.g., acetazolamide) are prohibited in competition.

## Conclusion

We had one goal in mind with this position paper: to protect athletes from potential harmful consequences of altitude training (i.e., primum non nocere). The current paper demonstrates that sleep during a typical altitude training protocol is impaired in an athletic population and that trait-like interindividual differences exist underlying these altitude-associated sleep impairments. The search for the hereditary and environmental factors underlying this trait is still in early stages, but already indicated a role for sex, polymorphisms in the TASK2/KCNK5, NOTCH4 and CAT gene, and pre-term birth. Furthermore, we reviewed current evidence indicating that physical activity can enlarge the altitude-associated sleep impairments. However, further research is necessary to elucidate the precise mechanisms and interactions. Hence, the present paper clearly demonstrates that sleep, besides iron deficiency and inflammation status, is an important factor in taking into account the intra- and interindividual variability in altitude training-associated responses. To further increase the effectiveness of altitude training by taking sleep into account, we advocate individualization, with a first step being screening for athlete’s responses to nocturnal hypoxia. Currently, polysomnography should be the first choice to evaluate an individual’s predisposition to altitude-associated sleep impairments. In addition, to further optimize the individualization of altitude training and predict who would benefit and who not, gene polymorphisms that have been found to play a role in the occurrence of altitude-associated sleep impairments should be determined in athletes.

## Author contributions

Both authors wrote the first draft of the manuscript, developed the position manuscript conception and design *via* open discussion, read, and approved the final manuscript.
